This article has been retracted.

# Subclinical Hypothyroidism and Its Association with Increased Cardiovascular Mortality

**DOI:** 10.1155/2017/7539735

**Published:** 2017-05-28

**Authors:** Alvaro Altamirano Ufion, Beenish Zulfiqar, Abdalla Hassan, Roshanak Habibi, Prajwal Boddu

**Affiliations:** ^1^Department of Internal Medicine, Advocate Illinois Masonic Medical Center, Chicago, IL 60657, USA; ^2^Department of Internal Medicine, Saint Francis Hospital, Evanston, IL 60202, USA; ^3^University of Texas, MD Anderson Cancer Center, Houston, TX 77030, USA

## Abstract

Thyroid hormones play an important role in regulating different metabolism functions and multiple organs' performance. Changes in the thyroid hormone axis can lead to profound effects on the stability of vital organs and systems, especially the cardiovascular system. Hypothyroidism is classified according to the clinical presentation as overt and subclinical. There is some evidence supporting the benefits of thyroxine hormone replacement for subclinical hypothyroidism on cardiovascular mortality outcomes. However, the clinical relevance of measuring and treating high thyroid-stimulating hormone (TSH) levels in newly diagnosed heart failure patients with preserved ejection fraction requires further study. In this report, we review the current evidence regarding the prognostic significance of subclinical hypothyroidism in heart failure patients with preserved ejection fraction.

## 1. Background

Thyroid hormones regulate different metabolism functions and multiple organs' performance. When the thyroid hormone axis is altered, it can lead to either hypo- or hyperthyroidism. Hypothyroidism presents clinically as overt or subclinical. Subclinical hypothyroidism is defined as the absence of symptoms with an increase in the levels of thyroid-stimulating hormone (TSH) with normal levels of free T3 and free T4. There is more information available about overt hypothyroidism than subclinical hypothyroidism. Overt hypothyroidism is well known to be associated with cardiovascular diseases, such as accelerated atherosclerosis and coronary artery disease. Both T3 and T4 seem to have beneficial effects in the cardiovascular system. T3 facilitates myocardial relaxation and decreases peripheral vascular resistance, whereas T4 replacement therapy helps improve hemodynamics in patients with subclinical hypothyroidism [1].

There is some evidence on the benefits of thyroid hormone replacement on cardiovascular mortality outcomes in subclinical hypothyroidism. However, the clinical relevance of measuring and treating high TSH levels in newly diagnosed heart failure patients with preserved ejection fraction requires further study. It has been proven that heart disease can alter thyroid hormone metabolism. Conversely, thyroid hormone dysfunction can result in altered ventricular contraction or relaxation along with compromised cardiac function. Thyroid dysfunction can act as a comorbid condition in favoring the onset/progression of HF [2].

## 2. Genetics

T4 constitutes the major circulating fraction of thyroid hormone in the human body. T4 is transformed by iodothyronine deiodinase into T3, the biologically active form responsible for the actual effects on target-end organs. T3 affects the cardiac muscle through two different mechanisms, genomic and nongenomic. Genomic effects are achieved through upregulation in the expression of genes involved in the production of structural proteins including sarco-/endoplasmic reticulum calcium-ATPase (SERCA) and cardiac myosin heavy chain [3]. Low thyroid hormone levels lead to decrease in levels of SERCA-2 activity, which controls the contraction and relaxation cycle through an adenosine 5′-triphosphatase (ATPase) with an affinity for calcium, leading to myocardial stiffness and eventually left ventricular diastolic dysfunction [4]. T3 binds to the thyroid hormone receptors in the nucleus. These nuclear receptors bind themselves to thyroid hormone responsive elements located in the promoter regions of specific genes. In the heart, these types of receptors have been identified as TR alpha-1, TR alpha-2, TR beta-1, and TR beta-2 [5]. They have different functions and can act as positive or negative regulators. For instance, the TR alpha-1 plays an important role in regulating some physiologic functions in the heart, while TR alpha-2 has an antagonistic physiological role by exerting negative regulatory effects on TR alpha-1 [6].

Thyroid hormones are involved in the regulation of hyperpolarization-activated cyclic nucleotide gated channels and proteins, and genes encoded in specialized pacemaker cells. Also, the angiotensin receptors in the smooth muscle cells of the vessels seem to be regulated by the T3 nuclear receptor [7]. Endothelial microparticles, which have been linked to endothelial injury and dysfunction, have also been found in patients with subclinical hypothyroidism, ischemic heart disease, and congestive heart failure. It has been observed that some of the involved genes encode for a specific type of protein that participates in the contraction of the heart muscle, such as alpha and beta (mentioned above), the sodium calcium exchanger, PLB, and the beta adrenergic receptor MHC. Once the expression of these genes is altered, there is a cascade of events where cardiac contractility, calcium cycling, and diastolic relaxation can be affected with the subsequent development of heart failure [8].

Patients with low levels of thyroid hormones seem to fall into a cycle where the low levels of thyroid hormones lead to heart failure. At the same time, heart failure can downregulate the signal of the thyroid hormones in the heart with a net effect of increase in overall mortality. If we combine this phenomenon with the effects on structures other than cardiac tissue, the overall mortality becomes significantly high [9]. One well-known example to mention is the association between higher levels of cholesterol in patients with hypothyroidism either overt or subclinical. As we know, hyperlipidemia is the main risk factor for coronary heart disease that ultimately can lead to heart failure. But more importantly, some studies suggest that more than 90% of patients with overt hypothyroidism and some patients with subclinical hypothyroidism can have derangements of the lipid profile, including low density lipoproteins (LDL) and apolipoprotein A. Treatment with thyroid hormones can lead to reversal of these derangements [10].

Another example is the histological changes that have been reported in some studies of animals with low levels of thyroid hormones. The animals have an accumulation of mucopolysaccharides in the heart, which can lead to impairment of the myocardium. This impairment is similar to the damage caused by other conditions that can lead to mucopolysaccharides accumulation in humans. Most of these are genetic conditions that eventually lead to heart failure; although strong evidence of this in humans actually lacks, there have been case reports evidencing this association [11].

One last example of this interaction between hypothyroidism and heart failure is that low T3 levels seem to have a direct correlation with the degree of left ventricular dysfunction and levels of NT-pro-beta natriuretic peptide, meaning that the lower the T3 levels, the more the left ventricular dysfunction and the higher the biological marker. However, this correlation does not exist with low levels of T4 or high levels of TSH. At the clinical level, there is correlation between low levels of T3 and idiopathic dilated cardiomyopathy [12].

This conclusion leads to an important question. If hypothyroidism is associated with increased mortality in heart failure and there is evidence suggesting that there is a benefit from replacing thyroid hormones, at what extent should we consider replacing them?

Regarding the question of whether subclinical hypothyroidism potentiates risk factors for heart failure, a study by Rodondi et al. found that the following risk factors have a statistically significant association with subclinical hypothyroidism: smoking, diabetes, presence of peripheral vascular disease, and high cholesterol levels. In the same study, there was a direct association with congestive heart failure, although the levels of thyroid-stimulating hormones (TSH) were more than 7 mIU/L to be statistically significant and the sample included only hospitalized patients [13].

## 3. Discussion

Clinical signs and symptoms poorly predict thyroid status, especially in the elderly population, and the diagnosis of subclinical hypothyroidism is based purely on biochemical grounds of elevated TSH with normal free thyroxine levels. As the diagnosis relies on an elevated level of TSH, identifying the upper limit of reference range is critical in defining subclinical hypothyroidism. Observations from the composite of all age groups in a large clinical trial designated a TSH level of 4.5 mIU/L as upper range of normal [14]. Various studies have suggested an increase in the incidence of subclinical hypothyroidism with aging [14–16]. However, normal TSH distributions shift toward higher concentrations with age, a consequence leading to overestimation of this diagnosis in the elderly [17]. A longitudinal cohort study looking at elderly patients did not find an association between subclinical hypothyroidism and cardiovascular or all-cause mortality, raising concern for treating mildly supranormal TSH levels based on currently recommended cut-off limits [18].

Patients with subclinical hypothyroidism represent a dimorphic population, either as prerunners of overt hypothyroidism with risk factors of thyroid disease or with an indolent form of disease with preserved thyroid function reserve [19]. A prospective study observed that up to 55% of subclinical hypothyroid patients with TSH levels more than 6 mIU/L eventually progressed to overt hypothyroidism over a 10-year follow-up period [20]. Clinical evidence of goiter and presence of anti-thyroid antibodies serve as predictive risk-stratifiers in determining progression toward overt hypothyroidism [20, 21].

The clinical importance of subclinical hypothyroidism in cardiovascular disease and mortality remains controversial, with most studies providing conflicting results. This may be explained by the selection of heterogenous patient populations, arbitrarily designated TSH reference limits in defining subclinical hypothyroidism, lack of stratification of study groups based on the degree of TSH elevation, varying study designs, and paucity of randomized controlled trials directly addressing patient-outcome relationships.

Despite extensive research, there still exists clinical uncertainty on various aspects surrounding thyroid-related cardiovascular disease. The most recent American College of Cardiology/American Heart Association guidelines for the diagnosis and management of heart failure recommend measuring thyroid function in all patients with newly diagnosed heart failure since it represents a potential reversible cause of cardiovascular disease. Nonetheless, no specific recommendations have been made with regard to the management of subclinical hypothyroidism in patients with heart failure [2].

Classification systems have been proposed that grade subclinical hypothyroidism based on severity assessment into grade 1 (TSH levels less than 10 mIU/L) or grade 2 (TSH more than 10 mIU/L) [22]. The natural history may differ significantly between the two groups with grade 2 category patients having higher cardiovascular events and higher rates of transition to overt hypothyroidism [23, 24]. A large prospective study involving an elderly population (>85 years) noted an association between grade 1 subclinical hypothyroidism and decreased all-cause mortality [25]. The higher cardiovascular mortality rates in group 2 subclinical hypothyroidism patients are related to known cardiovascular effects of thyroxine on heart function and metabolism. Cardiovascular alterations that occur in overt hypothyroidism have also been identified in subclinical hypothyroidism, effects varying only in the degree of derangement [26]. Of note, mouse model studies have demonstrated that serum thyroxine levels do not reflect cardiac tissue T4 levels in mild hypothyroidism, with cardiac tissue hypothyroidism occurring in the presence of normal serum thyroxine levels [27]. Increased systemic vascular resistance, arterial stiffness, and altered endothelial function have been associated with subclinical thyroid dysfunction. Enhanced cardiovascular risk has been also related to altered proatherogenic lipid profiles, a reversible condition with institution of levothyroxine replacement therapy [28]. The benefits of levothyroxine treatment on endothelial function and intima-media thickness have been well demonstrated in previous randomized trials [27, 29]. Whether or not these benefits lead to better clinical outcomes has yet to be determined.

In the Health Aging and Body Composition population-based study, the authors investigated the levels of thyroid-stimulating hormone affecting harmful cardiovascular consequences by following patients prospectively over 4 years. The study concluded that patients with TSH levels more than 7 mIU/L and more than 10 mIU/L had a hazard ratio of 2.58 and 3.26, respectively, for developing heart failure [30]. Another study conducted by Rodondi et al. of over 55,000 individuals demonstrated a positive correlation between the degree of TSH elevation and cardiovascular event rates and mortality [23]. Collet et al. collected data from 10 cohort studies which showed a hazard ratio for coronary heart disease related mortality of 1.24 and 1.21 for CHD events [31]. Several studies suggest that the cut-off level of TSH more than 10 mIU/L may be used to define a patient with subclinical hypothyroidism with an increased risk for cardiovascular events. The Cardiovascular Health Study performed echocardiogram routinely for 6 years in a cohort of patients to determine patients at risk for developing heart failure. It was found that patients with a TSH more than 10 mIU/L had higher risk of heart failure with low ejection fraction as compared to the population with normal thyroid function. Collet et al. also proved that the antibody status of an individual does not render higher risk for CHD since patients with clinical and subclinical hypothyroidism may or may not have positive antibodies [32].

The cardiac-ankle vascular index, an indicator of arteriosclerosis, has been studied in subclinical hypothyroidism and increased index values have been associated with elevated beta natriuretic peptide (BNP) levels, reflecting the effect of decreased tissue T3 levels in the alteration of the ventricular and arterial wall pressure dynamics [33]. While many studies describe the relation between heart disease and overt hypothyroidism, one study suggested that dilated cardiomyopathy is associated with subclinical hyperthyroidism as opposed to subclinical hypothyroidism [34].

It has also been noted that the levels of T3 correlate with the functional level according to their New York Heart Association Class (NYHA) and that lower hormone levels are associated with higher NYHA classification, making it a predictor of mortality in classes III and IV of the NYHA [35, 36]. In patients with heart failure with preserved ejection fraction, a study showed that up to 22% of these patients had altered thyroid function with low T3 levels [35]. However, available evidence, based on current literature, is still contradicting in certain groups of patients. In a study conducted on patients with heart failure and reduced ejection fraction, neither subclinical hyperthyroidism nor hypothyroidism was found to be significant prognostic factors [37].

## 4. Clinical Perspectives

The association between cardiovascular disease and subclinical hypothyroidism, though significant, is reversible with thyroxine hormone replacement, as reflected by improvement, or reversal in some of the components such as diastolic dysfunction and carotid artery intima- media thickness (a marker of subclinical atherosclerosis) [38, 39]. In 2005, a consensus panel from three recognized organizations such as the American Association of Clinical Endocrinologists, the American Thyroid Association, and the Endocrine Society recommended against replacing thyroid hormones if TSH is <10, but that treatment was reasonable in patients with subclinical hypothyroidism if TSH was >10 [40]. Current clinical practice guidelines recommend treating subclinical hypothyroid patients with TSH levels greater than 10 mIU/L [41]. Thyroxine replacement for TSH levels less than 10 mIU/L should be patient specific and tailored based on age characteristics and clinical hypothyroidism symptoms. More studies need to be conducted to determine the appropriateness of thyroxine replacement by identifying a specific high-risk subset of subclinical hypothyroid patients, including those likely to progress to overt hypothyroidism [40]. Select patients with heart failure would benefit from thyroid hormone replacement if they are discovered to have subclinical hypothyroidism. This therapeutic benefit is more so in patients with heart failure with preserved ejection fraction, a relatively less well-studied population.

## 5. Conclusion

To summarize, we may conclude that hypothyroidism and its subclinical counterpart have prognostic implications in patients with heart failure due to its association with increased cardiovascular mortality. Since there exists some evidence of a causal relationship, it may seem appropriate to perform a basic cardiac work-up like an echocardiogram to assess for subclinical systolic and diastolic dysfunction as part of initial evaluation of hypothyroid patients. Evidence of cardiac dysfunction may facilitate the determination of appropriateness of thyroxine replacement therapy in subclinical hypothyroidism.

## Abbreviations

TSH: Thyroid-stimulating hormone
T3: Triiodothyronine
T4: Thyroxine or Tetraiodothyronine
SERCA: Sarco-/endoplasmic reticulum calcium-ATPase
ATPase: Adenosine 5′-triphosphatase
NYHA: New York Heart Association.
